The article "Exploration of Potential Biomarkers and Immune Landscape for Hepatoblastoma: Evidence from Machine Learning Algorithm" was retracted in 2023. Reasons: signs of a paper mill; suspected computer-generated content; unreliable results or conclusions; lack of ethics approval or compliance.

# Exploration of Potential Biomarkers and Immune Landscape for Hepatoblastoma: Evidence from Machine Learning Algorithm

**DOI:** 10.1155/2022/2417134

**Published:** 2022-07-31

**Authors:** Peng Zhou, Shanshan Gao, Bin Hu

**Affiliations:** ^1^Department of Pediatric, Maternal and Child Health Hospital, Zibo, China; ^2^Department of Ultrasound, Zibo Forth People's Hospital, Zibo, China

## Abstract

This study aimed to investigate the immune landscape in hepatoblastoma (HB) based on deconvolution methods and identify a biomarkers panel for diagnosis based on a machine learning algorithm. Firstly, we identified 277 differentially expressed genes (DEGs) and differentiated and functionally identified the modules in DEGs. The Kyoto Encyclopedia of Genes and Genomes (KEGG) analysis and GO (gene ontology) were used to annotate these DEGs, and the results suggested that the occurrence of HB was related to DNA adducts, bile secretion, and metabolism of xenobiotics by cytochrome P450. We selected the top 10 genes for our final diagnostic panel based on the random forest tree method. Interestingly, TNFRSF19 and TOP2A were significantly down-regulated in normal samples, while other genes (TRIB1, MAT1A, SAA2-SAA4, NAT2, HABP2, CYP2CB, APOF, and CFHR3) were significantly down-regulated in HB samples. Finally, we constructed a neural network model based on the above hub genes for diagnosis. After cross-validation, the area under the ROC curve was close to 1 (AUC = 0.972), and the AUC of the validation set was 0.870. In addition, the results of single-sample gene-set enrichment analysis (ssGSEA) and deconvolution methods revealed a more active immune responses in the HB tissue. In conclusion, we have developed a robust biomarkers panel for HB patients.

## 1. Introduction

The most prevalent pediatric liver tumor is hepatoblastoma (HB), which mostly affects children under the age of four. HB is an uncommon pediatric cancer with an annual incidence of 1.5 cases per million [1]. Up to 80% of all patients diagnosed with cancer survive thanks to complete surgical resection and treatment. Unfortunately, immunosuppression may have long-term negative effects in survivors [2]. The absence of excellent early diagnosis techniques is the primary cause of poor prognosis. Nowadays, clinicians identify the condition based on clinical signs, imaging, and methotrexate levels. Due to the many sources of AFP in patients, the sensitivity and specificity are insufficient [3]. A case reported that five individuals with normal AFP levels were diagnosed with HB [4]. As a result, novel and robust biomarkers must be discovered in order to create effective diagnostic and therapeutic procedures for HB patients.

The article "Exploration of Potential Biomarkers and Immune Landscape for Hepatoblastoma: Evidence from Machine Learning Algorithm" was retracted in 2023. Reasons: signs of a paper mill; suspected computer-generated content; unreliable results or conclusions; lack of ethics approval or compliance.

With the development of high-throughput sequencing technology, more and more aberrantly expressed mRNAs have been identified in HB [5–7]. Moreover, the elevated N6-methyladenosine alteration in HB represents a carcinogenic pathway [8]. Several studies have also found that various genes, such as zinc finger antisense 1 [9] and TUG1 [10], are involved in proliferation, apoptosis, and glutaminolysis. Importantly, the liver has specific histology and microenvironment that controls tumor growth and therapeutic outcome: dual blood supply, vascularization of porous blood sinuses, and the presence of different mesenchymal cells [11]. The liver exhibits a specific immune response to tumor cells, which correlates with poor responsiveness to immunotherapy [12]. Therefore, assessing the altered immune microenvironment in HB could provide a more reliable therapeutic strategy for patients. Because of the various analytical methodologies, experimental methods, and sample sizes used in the investigations, the findings are debatable. As a result, more bioinformatics investigations from public databases might help to reveal the immune landscape and novel biomarkers panel in HB patients.

The study aimed to reveal reliable differentially expressed genes in HB using datasets from the Gene Expression Omnibus (GEO) database. Subsequently, we discovered hub genes using machine learning methods and utilized them to build a neural network for diagnosis. In addition, we studied the status of the immune microenvironment as well as hundreds of tumor microenvironment-related pathways in depth. We hope that the biomarkers panel in this study will lead to the development of novel diagnostic and prognostic for HB patients.

## 2. Methods

### 2.1. Datasets and Data Preprocessing

RNA-seq datasets were downloaded from the GEO database [13]: GSE131329 datasets based on the GPL6244 platform (14 noncancerous liver tissue samples and 53 HB samples) and GSE133039 datasets based on the GPL16791 platform (32 noncancerous liver tissue samples and 31 HB samples). The GSE131329 datasets were defined as screening sets, and the GSE133039 dataset was used as an external validation set.

### 2.2. Screening of Biomarkers Panel

Differentially expressed genes (DEGs) were identified in the screening set using the “limma” package in R software [14]. We selected|log  2 fold change FC| > 2and adj.*P*.value < 0.05 as criteria. The random forest tree [15] (the optimal number of variables in the binomial tree in the node is 6, the optimal number of trees contained in the random forest is 2000, and the top10 genes in importance analysis were selected) was used to identify 10 hub genes as final biomarkers panel.

The article "Exploration of Potential Biomarkers and Immune Landscape for Hepatoblastoma: Evidence from Machine Learning Algorithm" was retracted in 2023. Reasons: signs of a paper mill; suspected computer-generated content; unreliable results or conclusions; lack of ethics approval or compliance.

### 2.3. Neural Network

We selected the screening set for neural network model training, and the validation set was tested using the same process. A neural network model based on a biomarkers panel was constructed using the “neuralnet” package [16] in R software after normalizing the data to the maximum and minimum values. Subsequently, four hidden layers were set as model parameters, and the classification model of the disease (HB or normal) was constructed by the obtained gene weight information. It is worth noting that the sum of the product of the weight score and the expression level of significant genes is used as the disease classification score. In addition, we performed a 10fold validation of the model results. Finally, the “pROC” package [17, 18] in R software was used to calculate the AUC value in classification performance.

### 2.4. Identification of Hub MCODEs in Protein-Protein Network and Enrichment Analysis

We used metascape online tools [19] to construct hub MCODEs in DEGs and annotated biological functions in each hub MCODEs. GO enrichment analysis [20] is a commonly used bioinformatics method for comprehensive information, including biological process, cellular component, and molecular function. In addition, KEGG pathway enrichment analysis [21] is widely used to explore biological mechanisms and functions. We selected q value and *P* value < 0.05 as criteria.

### 2.5. Analysis of Tumor Immune Microenvironment

We used the single-sample gene-set enrichment analysis (ssGSEA) to quantify the tumor immune microenvironment (TIME) associated pathways in each tissue sample. The “IOBR” package [22] was used to download and analyze the gene sets of “TME-associated pathways.” In addition, xCell, EPIC, MCPcounter, and timer algorithms were used to analyze the immune infiltration levels of cells in TME. The heatmap diagram was used to compare the differences between immune cells and TME-associated pathways in different tissues.

### 2.6. Cell Lines and Quantitative Real-Time PCR (qRT-PCR)

The HB cell lines (SMMC-7721) and the normal human hepatic cell line (L02) were cultured in 10% FBS DMEM medium in an environment of 5% CO2 and 37°C [23]. Primer sequences are summarized in previous studies, including TRIB1 [24], MAT1A [25], SAA2-SAA4 [26], NAT2 [27], HABP2 [28], CYP2CB [29], APOF [30], and CFHR3 [31]. Detailed experimental procedures are described in our previous publications [32, 33].

### 2.7. Statistics

We implemented all statistical analyses with R version 4.1.1. Wilcox test was used to screen infiltrating immune cells or scores of TME-associated pathways with statistically significant. *P* < 0.05 was considered statistically significant.

The article "Exploration of Potential Biomarkers and Immune Landscape for Hepatoblastoma: Evidence from Machine Learning Algorithm" was retracted in 2023. Reasons: signs of a paper mill; suspected computer-generated content; unreliable results or conclusions; lack of ethics approval or compliance.

## 3. Results

### 3.1. Differential Expression Genes in Different Samples

We performed differentially expressed genes analysis in the screening set and finally identified 277 DEGs, and the heatmap shows the top30 DEGs (Figure 1(a)). The volcano plot demonstrated 90 up-regulated genes as well as 187 down-regulated genes (Figure 1(b)).

### 3.2. Hub Modules in DEGs Network

Considering the interactions between DEGs, we differentiated and functionally identified the modules in 277 genes (Figure 2). In the red module, it was mainly composed of CYP and UGT family genes and was associated with DNA adducts, biological oxidations, and xenobiotic processes. In the blue module, it was mainly composed of H2BC5, AR, SDS, H2BC3, and H2AC13; the module was associated with activated PKN1 stimulating transcription of AR-regulated genes, condensation of prophase chromosomes, and HDACs deacetylate histones. Finally, in the red module, BMP4, GPC3, NOTUM, CP, MATN3, AFP, ORM1, TGFB2, SERPINE1, HGF, ORM2, and HRG derived from the module and was associated with platelet degranulation.

### 3.3. Enrichment Analysis

We revealed that 277 DEGs were significantly associated with HB in differentially expressed genes analysis. The Kyoto Encyclopedia of Genes and Genomes (KEGG) analysis was used to annotate these DEGs (Figure 3(a)). Similar to the results enriched in the hub modules, the results of KEGG analysis also showed that DNA adducts, bile secretion, and metabolism of xenobiotics by cytochrome P450 played a key role in the occurrence of HB. The GO analysis showed that the xenobiotic metabolic process, long-chain fatty acid metabolic process, and olefinic compound metabolic process were associated with HB (Figure 3(b)).

### 3.4. Construction of Biomarkers Panel

The random forest tree method was used to sort the weights of all DEGs (Figures 4(a) and 4(b)). Selecting the top 10 genes for our final diagnostic panel, the heatmap showed the expression landscape in different tissues. Interestingly, TNFRSF19 and TOP2A were significantly down-regulated in normal samples, while other genes (TRIB1, MAT1A, SAA2-SAA4, NAT2, HABP2, CYP2CB, APOF, and CFHR3) were significantly down-regulated in HB samples (Figure 4(c)).

### 3.5. Construction of the Artificial Neural Network Model

We built an artificial neural network model based on the “neuralnet” package. The min-max method [0, 1] was chosen for normalizing the data segment and scale data, and then, the neural network was trained to normalize the maximum and minimum values of the data, the number of hidden layers was set to 5 before starting the computation, and the parameter for the number of neurons was set to 6. The neural network model, including a total of 4123 steps, had been carried out in the training set (Figure 5(a)). In order to evaluate the results of the neural network model more effectively, we choose the method of 10 cross-validations. After cross-validation, the area under the ROC curve is close to 1 (AUC = 0.972), indicating robustness (Figure 5(b)). It was worth noting that in the validation set, the AUC of the neural network model was 0.87 (Figure 5(c)).

The article "Exploration of Potential Biomarkers and Immune Landscape for Hepatoblastoma: Evidence from Machine Learning Algorithm" was retracted in 2023. Reasons: signs of a paper mill; suspected computer-generated content; unreliable results or conclusions; lack of ethics approval or compliance.

### 3.6. The Landscape of Infiltrating Immune Cells and TME-Associated Pathways

We used the four deconvolution methods to characterize the immune cell pattern in HB. In the EPIC algorithm, the proportions of B cells and macrophage cells were significantly decreased in the tissues of HB patients. However, the proportions of CD8 T cells, CAFs, and endothelial cells were significantly increased in the tissues of HB patients (Figure 6(a)). In the MCPcounter algorithm, only the proportions of CD8 T cells were significantly decreased in the tissues of HB patients (Figure 6(b)). In the TIMER algorithm, four different types of immune cells also differed significantly between the two groups (Figure 6(c)). Finally, both the xCELL algorithm (Figure 6(d)) with more results and the enrichment results of TME-related pathways (Figure 7) showed a more active immune response in the HB tissue. The above results showed that the occurrence and development of HB were closely related to TME.

### 3.7. Quantitative Real-Time PCR (qRT-PCR)

For validating the expression of hub genes, HB cell lines (SMMC-7721) and L02 (L02) were used to conduct a qRT-PCR assay. In the validation ofTRIB1, MAT1A, SAA2-SAA4, NAT2, HABP2, CYP2CB, APOF, and CFHR3, the expression of SMMC-7721 was higher than that of L02 (Figure 8). The above results suggested that these hub genes may be potential oncogenic genes, but further experimental verification was still needed.

## 4. Conclusion

We developed the HB diagnostic classification model employing a random tree and 10 hub genes in this study. We also used an independent dataset to test the classification efficiency based on an artificial neural network. As a result, the model might aid with HB diagnosis. We also used GO and KEGG analyses to discover that the DEGs were mostly involved in DNA adducts, bile secretion, metabolism of xenobiotics by cytochrome P450, xenobiotic metabolic process, long-chain fatty acid metabolic process, and olefinic compound metabolic process. We studied the status of the TME as well as hundreds of TME-related pathways in depth. Finally, all algorithms and the enrichment results of TME-related pathways showed a more active immune response in the HB tissue.

The article "Exploration of Potential Biomarkers and Immune Landscape for Hepatoblastoma: Evidence from Machine Learning Algorithm" was retracted in 2023. Reasons: signs of a paper mill; suspected computer-generated content; unreliable results or conclusions; lack of ethics approval or compliance.

The 10 genes in our panel were as follows: TNFRSF19, TOP2A, TRIB1, MAT1A, SAA2-SAA4, NAT2, HABP2, CYP2CB, APOF, and CFHR3. Unfortunately, current basic research in HB had not addressed the above-mentioned genes in depth. Therefore, the discussion focused on the function of 10 genes themselves and their important role in the development of hepatocellular carcinoma (HCC). TNFRSF19 is a type I cell surface receptor protein that belongs to the tumor necrosis factor receptor (TNFR) superfamily [34]. TNFRSF19 is mainly expressed in the brain and prostate, with modest expression seen in the heart, spleen, colon, kidney, lung, liver, and peripheral blood lymphocytes [35]. According to recent research. In glioblastoma multiforme (GBM), TNFRSF19 expression is highly increased, and it enhances glioma cell motility and invasion in vitro [36]. TNFRSF19, on the other hand, has been shown to operate as a negative regulator of WNT signaling, and suppression of TNFRSF19 expression has been linked to a reduced overall survival rate [37]. TNFRSF19 expression was shown to be considerably lower in HCC tissue than in normal tissue in one investigation. Reduced TNFRSF19 led to increased proliferation and invasion of HCC cells, implying that TNFRSF19 may function as a tumor suppressor [38]. The TOP2A can encode a DNA topoisomerase that is responsible for controlling and altering DNA topology during transcription [39]. In addition, TOP2A expression in different cancers is considered to be a favorable prognostic biomarker for predicting cancer progression and recurrence, and it can also serve as a risk factor for low survival [40]. In HCC, several studies have shown TOP2A up-regulation [41, 42]. TRIB1 has a conserved motif similar to the catalytic domain of serine/threonine kinases but lacks the ATP-binding or kinase catalytic domain [43]. TRIB1 acts as a scaffold or bridging protein, promotes the degradation of target proteins, and regulates several important signaling pathways [44]. Due to physical interactions, TRIB1 suppresses the tumor suppressor gene p53, the most commonly mutated gene in HCC, which plays a key role in many cancers [45]. Mammals have three different forms of MAT (MATI, MATII, and MATIII), encoded by two different genes (MAT1A and MAT2A). MAT in the liver and extrahepatic tissues is the product of two genes, MAT1A and MAT2A, respectively [46]. MAT1A is a strong prognostic indicator for HCC, and data from HCC patients with reduced MAT1A suggest that the RETOME pathway may be involved in HCC tumorigenesis [47]. However, the remaining genes are equally poorly studied in HCC, which reminds us of the gaps in the field of HB-related hub gene research. In conclusion, we have developed a robust biomarkers panel for HB patients.

The article "Exploration of Potential Biomarkers and Immune Landscape for Hepatoblastoma: Evidence from Machine Learning Algorithm" was retracted in 2023. Reasons: signs of a paper mill; suspected computer-generated content; unreliable results or conclusions; lack of ethics approval or compliance.

## 5. Conclusions

We studied the status of the immune microenvironment as well as hundreds of tumor microenvironment-related pathways in-depth and revealed more active immune responses in the HB compared to normal tissues. Moreover, we hope that the biomarkers panel will lead to diagnostic development for HB patients.

## Figures and Tables

**Figure 1:** Differential expression analysis. (a) The heatmap of differential expression genes in screening dataset. (b) The volcano plot of differential expression genes in the screening dataset.

**Figure 2:** Hub modules from metascape online tools.

**Figure 3:** Enrichment analysis. (a) The terms of KEGG enrichment analysis. (b) The terms of GO enrichment analysis.

**Figure 4:** Differential expression analysis. (a) The process of constructing random forest trees. (b) Ranking of gene importance. (c) The heatmap of the top 10 genes in the screening dataset.

**Figure 5:** Construction and validation of the artificial neural network model. (a) Construction of the artificial neural network model. (b) ROC curve in screening dataset. (c) ROC curve in the validation dataset.

**Figure 6:** The landscape of infiltrating immune cells is based on 4 deconvolution methods. (a) Heatmap of immune cell content in different tissues (EPIC algorithm). (b) Heatmap of immune cell content in different tissues (MCPcounter algorithm). (c) Heatmap of immune cell content in different tissues (TIMER algorithm). (d) Heatmap of immune cell content in different tissues (xCELL algorithm).

**Figure 7:** The landscape of TME-associated pathways.

**Figure 8:** qRT-PCR validation.

## Data Availability

Data are available at the GEO database (https://www.ncbi.nlm.nih.gov/geo/).
